# Effect of Painless Rehabilitation Nursing for Hip Replacement Patients

**DOI:** 10.1155/2022/5164973

**Published:** 2022-06-11

**Authors:** Xiaona Zhao, Ru Bai, Jing Yang

**Affiliations:** ^1^Yuncheng Central Hospital, Yuncheng, China; ^2^Yuncheng Vocational and Technical University, Yuncheng, China; ^3^Nursing College of Shanxi Medical University, Shanxi, China

## Abstract

**Objective:**

To analyze the effect of painless rehabilitation nursing for hip replacement patients.

**Method:**

124 elderly patients who underwent total knee arthroplasty in our hospital from June 2019 to June 2020 were selected as study subjects. They were randomly divided into observation group and control group. The control group was given routine nursing care, and the observation group was given painless rehabilitation care on the basis of the control group. Knee circumference, knee pain, knee function, agitation and sleep duration were recorded and compared between the two groups.

**Results:**

The changes of knee circumference diametral in both groups were significantly decreased at 1, 3 and 7 days after operation; The changes of knee circumference diametral in the observation group were significantly smaller than those in the control group at 3,7 days after operation (*P <0.05*). VAS (Visual Analogue Scale) scores at 1, 3 and 7 d after operation were significantly decreased in both groups; The score of the observation group was significantly lower than that of the control group, and the difference was statistically significant (*P <0.05*). HSS (Hospital for special surgery) scores increased significantly in both groups at 1 week, 1 month, 3 months and 6 months after operation. All the comparisons were statistically significant (*P <0.05*); HSS scores of observation group were significantly higher than control group at 1 week, 1 month, 3 months and 6 months after surgery. The difference was statistically significant (*P <0.05*). The agitation rate of the observation group was lower than that of the control group (*P <0.05*). Compared with the control group, the sleep time of observation group increased significantly in each period, with statistically significant difference (P <0.05).

**Conclusion:**

Perioperative painless rehabilitation nursing interventions for patients with hip replacement could significantly relieve swelling and pain, it was helpful for the patients to recover the function of knee joint after operation and worthy of clinical application.

## 1. Introduction

In clinic, femoral neck fracture usually occurs in the elderly. Hip replacement is mainly used in the elderly patients with femoral neck fracture in clinical, mainly for the elderly patients over 50 years old.Due to the inability of the affected limb to walk with weight after fracture, it needs to stay in bed for a long time, but it is prone to serious bed complications such as bedsore, accumulated pneumonia, urinary tract infection and lower extremity deep venous thrombosis, which is difficult to care [1].the treatment effect of acetabular degeneration, articular ankylosis, femoral head necrosis, femoral neck fracture and other symptoms is good, which can effectively restore the patient's hip function [2]. The operation process of total hip arthroplasty is convenient and operable, and the incidence of postoperative adverse reactions is relatively low and the safety factor is high [3]. Hip arthroplasty is the most effective method for the treatment of hip disease and femoral neck fracture. This operation is to place a metal prosthesis similar to human bone and joint into the damaged joint surface. The ultimate purpose of hip arthroplasty is to restore joint function and eliminate pain, but the recovery of joint function after arthroplasty is closely related to patients' postoperative rehabilitation exercise [4]. Due to the poor physical quality of the elderly patients, the incidence of postoperative complications is higher. Therefore, how to perform effective analgesia for patients with hip joint disease is of great significance [5, 6]. Early rehabilitation nursing intervention as soon as possible after the recovery of patients' consciousness can not only improve their psychological state, but also enhance the patients' attention to postoperative rehabilitation exercise, effectively alleviate their pain and create conditions for the smooth progress of follow-up rehabilitation exercise [7]. Studies have shown that painless rehabilitation care has a more prominent effect in preventing postoperative pain and can promote faster recovery of patients [8, 9].

To analyze the effect of painless rehabilitation nursing for hip replacement patients. 124 elderly patients who underwent total knee arthroplasty in our hospital from June 2019 to June 2020 were selected as study subjects. The indexes of knee circumference diameter and knee pain were observed 1, 3 and 7 days after operation; The indexes of knee function、agitation situation and sleep time were observed 1 week, 1 month and 3 months after operation. The application effect of painless rehabilitation nursing for hip replacement patients was discussed by analyzing the data of the above five observation indexes. The rest of our paper consists as section-2 illustrates materials and methods that we have used during our research work, section-3, makes a comparative analysis of the two groups of cases, section-4 is based on discussing and finally, we conclude our work in section-5.

The detailed research content is as follows:

## 2. Materials and Methods

### 2.1. General Information

According to the following exclusion criteria and inclusion criteria, 124 elderly patients who underwent total knee arthroplasty in our hospital from June 2019 to June 2020 were selected as study subjects.

#### 2.1.1. Inclusion Criteria

1. No cognitive or mental disorders
2. Meeting the relevant indications for hip replacement [10];
3. American Association of Anesthesiologists (ASA) grade I ~ III [11].

#### 2.1.2. Exclusion Criteria

1. Patients with malignant tumors, cognitive impairment, contraindications to anesthesia and incomplete clinical data
2. Preoperative analgesic drugs were used
3. Severe heart and lung dysfunction
4. Other persons who were not suitable to be enrolled

124 cases were divided into control group and observation group to be grouped by lot: In the control group, there were 62 cases, including 39 males and 23 females, the average age was (74.29 ± 3.35) between 66 and 85 years old, the body mass was 56~69 kg, with an average weight of (62.25 ± 2.36) kg. In the observation group, there were 62 cases, including 33 males and 29 females, the average age was (73.24 ± 3.32) between 64 and 85 years old, the body mass was 55~72 kg, with an average weight of (62.21 ± 2.65) kg. Participants and their families were informed, and baseline information remained homogeneous between groups (P > 0.05). The grouping details are shown in Table 1.

### 2.2. Methods

During the perioperative period, the observation group adopted conventional nursing, namely preoperative examination under the guidance of the responsible nurse, formulation of personalized diet plan, preoperative psychological counseling, and intraoperative cooperation with the attending physician to complete the operation. Paying close attention to the changes of vital signs, follow the doctor's advice for routine treatment and resume knee function exercise. In the control group, the following measures were added to the perioperative nursing of the observation group: Preoperative evaluation; Pain education; Pain management; Pain care; Rehabilitation; Nutritional support; Psychological support. Details of the above measures are as follows:

1. Preoperative evaluation. After admission, the patient's physical condition was comprehensively evaluated based on the patient's health status and examination results to ensure the patient's tolerance during the operation, and the patient's vital signs were monitored in detail and make detailed paper records. Ensure that patients receive adequate nutritional support, psychological preparation and adequate preoperative preparation
2. Pain education. For different fear levels of pain, publicity materials related to painless care are posted in the ward, pain education manuals are distributed to patients, and psychological communication is carried out with patients to help patients deepen their understanding of pain
3. Pain management. For preoperative analgesia, celecoxib (200 mg) was given to the patient 3 days before the operation, twice a day, for 1 week after the operation. During the operation, femoral nerve combined with sciatic nerve block anesthesia was performed on the basis of general anesthesia. Attention was paid to keep warm during the operation, and intraoperative infusion volume was controlled. After surgery, when the patient returned to the ward, multimodal postoperative pain control was performed, such as parecoxib intramuscular injection [12] (40 mg), 2 times/d, continuous 3 days; continuous ice application for 48 hours; The intravenous self-controlled analgesia pump was used continuously for 48 hours
4. Pain care. Instructing patients to keep warm and keep the surgical site clean to prevent infection, patients with severe pain could be treated with central analgesics or a combination of non-steroidal anti-inflammatory analgesics [13] as prescribed by the doctor. For the pain caused by the postoperative incision and tight dressing, corresponding treatment could be given according to the specific situation, and the patient's pain symptoms should be evaluated in time. Letting patients relax their muscles by closing their eyes, meditation, deep breathing, sighing, and yawning to achieve the effect of pain relief. At the same time, various physical therapy methods such as cold compresses, ice compresses, hot compresses, appropriate relaxation of bandage and slight massage various physical treatment methods were used to relieve pain
5. Rehabilitation. Within 1 week after the operation, the patient was mainly manifested as local swelling and pain, and appropriate isometric exercises could be performed to help restore the original physiological function of the limb. Two weeks after the operation, the main symptoms were inflammation disappeared, callus formation and fracture end stability. There were moderate amount on the basis of muscle contraction exercise, gradually moving up and down joints. Prevent muscle atrophy
6. Nutritional support. If the patient had no symptoms of abdominal pain or abdominal distension 1 day after the operation, patient could eat an appropriate amount of fat-free or semi-liquid food. Under the guidance of the medical staff, patients were instructed to eat more light food which was easy to digest and rich in high quality protein, and eat more fresh vegetables and fruits
7. Psychological support. Guide patients to correctly face the pain caused by operation after operation; Face the difficulties encountered in recovery with a positive attitude; Provide psychological support for patients' family members in helping patients recover. Actively prevent patients from mental diseases such as depression and mania

Both groups were followed up for 5 months by telephone or outpatient follow-up, the follow-up period was from July 2020 to November 2020. And the recovery of knee joint function was recorded in detail.

### 2.3. Obvervational Index

Knee circumference, knee pain, knee function, agitation and sleep duration were compared between the two groups.

(1) Knee circumference (1, 3, 7d postoperatively). Preoperative and postoperative circumference of affected knee joint 1,3,7 d were measured by scale method. To improve the measurement accuracy, gentian violet could be used to mark the upper edge of the skeleton and marked the upper edge of the skeleton at 2 cm. A soft tape measure was used to measure the circumference (mm) of the knee joint at 2 cm above the upper margin of the skeleton. The change of knee circumference diameter (mm) = the circumference diameter on the n day after surgery - the circumference diameter before surgery, in which n was 1, 3, 7d
(2) Knee pain (1,3,7 d postoperatively). VAS Scale [14] (Visual Analogue Scale. This method is sensitive and comparable. Draw a 10 cm horizontal line on the paper. One end of the horizontal line is 0, indicating no pain; The other end is 10, indicating severe pain; The middle part indicates different degrees of pain.) was used to score the knee pain of the patients. 0 ~ 3 points: the patient had mild pain but can tolerate; 4 ~ 6 points: the patient's pain was more obvious, but could endure, if necessary, oral analgesic drugs; 7 ~ 10 points: The patient had more intense pain, pain severe unbearable
(3) Knee function. HSS Scale [15] (Hospital for Special Surgery. The knee scoring system was proposed by the American Hospital for Special Surgery in 1976 to evaluate the preoperative and postoperative function of the knee. The main evaluation indexes include: pain, function, joint range of motion, muscle strength, knee flexion deformity and knee instability.) was used to score the knee joint function of the patients. There were 6 items including pain (30 points), function (22 points), activity (18 points), muscle strength (10 points), flexion deformity (10 points) and stability (10 points), and the scoring range was 0 ~ 100 points
(4) Agitation condition. SAS (Sedative-Agitation Scale-A psychological scale used to measure the severity of anxiety and its changes during treatment. It is mainly used for efficacy evaluation, not for diagnosis.) [16] was used to evaluate, according to the level of normal: in a quiet state, could easily wake up, and obeyed the command; Mild agitation: body agitation, emotional anxiety, after verbal reminder could keep quiet; Moderate agitation: repeated verbal reminders or protective restraint; Severe agitation: The patient was aggressive and struggles violently
  (1) $$\begin{array}{c} \text{Agitation Rate}=\left(\text{Mild Agitation}+\text{Moderate Agitation}+\text{Severe Agitation}\right)/\text{total number}\times 100\%. \end{array}$$
(5) Sleep time. The sleep time of the patients before, after and 1d after the operation was recorded

### 2.4. Statistical Method

SPSS 19.0 statistical software was used for calculation and analysis. The measurement data were expressed as x ± s, t test was used for measurement data. Enumeration data was expressed in cases (%), x^2^ test was used for counting data. *P <0.05* was considered statistically significant.

## 3. Results

### 3.1. Results of Knee Circumference Diameter

The changes of knee circumference diametral in both groups were significantly decreased at 1, 3 and 7 days after operation; The changes of knee circumference diametral in the observation group were significantly smaller than those in the control group at 3,7 days after operation (*P <0.05*). Results of knee circumference diameter was shown in Table 2:

### 3.2. Results of Knee Pain

VAS (Visual Analogue Scale) scores at 1, 3 and 7 d after operation were significantly decreased in both groups; The score of the observation group was significantly lower than that of the control group, and the difference was statistically significant (*P <0.05*). Results of knee pain was shown in Table 3:

### 3.3. Results of Knee Function

HSS (Hospital for special surgery) scores increased significantly in both groups at 1 week, 1 month, 3 months and 6 months after operation. All the comparisons were statistically significant (*P <0.05*); HSS scores of observation group were significantly higher than control group at 1 week, 1 month, 3 months and 6 months after surgery. The difference was statistically significant (*P <0.05*). Results of knee function was shown in Table 4:

### 3.4. Result of Agitation Situation

The agitation rate of the observation group was lower than that of the control group (*P <0.05*). Result of agitation situation was shown in Table 5:

### 3.5. Result of Sleep Time

Compared with the control group, the sleep time of observation group increased significantly in each period, with statistically significant difference (*P <0.05*). Result of sleep time was shown in Table 6:

## 4. Discussion

For patients undergoing hip replacement operation, getting out of bed as soon as possible after surgery can effectively prevent deep vein thrombosis of the lower extremities [17]. Lower extremity deep venous thrombosis is the main complication of hip arthroplasty, but postoperative pain leads most patients to dread early functional exercise, which leads to a series of complications [18]. Pain affects the mood, confidence and expectation of future healthy life of patients undergoing hip arthroplasty. Therefore, pain is an important index that should be considered in postoperative nursing of patients undergoing hip arthroplasty [19]. Studies have shown that good postoperative analgesia care can shorten the recovery time of patients and reduce the risk of postoperative complications [20]. The painless management system has been applied well in many departments. With the continuous improvement of medical standards in recent years, people's demand for quality of care has also been rising, and pain care has gradually attracted attention [21]. Traditional Chinese medicine physiotherapy, related gymnastics and targeted limb movements can have a certain effect on the postoperative rehabilitation of patients undergoing hip arthroplasty. Clinical studies have shown that effective psychological intervention and pain care can significantly reduce patients' negative emotions and pain response [22]. Continuous psychological counseling for patients after operation can alleviate the anxiety or depression of patients and contribute to the rehabilitation of patients [23]. Therefore, painless rehabilitation nursing of patients undergoing hip arthroplasty is one of the hotspots of orthopaedic nursing.

This study showed that the changes of knee circumference diametral in both groups were significantly decreased at 1, 3 and 7 days after operation; The changes of knee circumference diametral in the observation group were significantly smaller than those in the control group at 3,7 days after operation (*P <0.05*). VAS (Visual Analogue Scale) scores at 1, 3 and 7 d after operation were significantly decreased in both groups; The score of the observation group was significantly lower than that of the control group, and the difference was statistically significant (*P <0.05*).HSS scores increased significantly in both groups at 1 week, 1 month, 3 months and 6 months after operation. All the comparisons were statistically significant (*P <0.05*); HSS scores of observation group were significantly higher than control group at 1 week, 1 month, 3 months and 6 months after surgery. The difference was statistically significant (*P <0.05*). The agitation rate of the observation group was lower than that of the control group (*P <0.05*). Compared with the control group, the sleep time of observation group increased significantly in each period, with statistically significant difference (*P <0.05*).

## 5. Conclusion

To sum up, the perioperative painless rehabilitation nursing interventions for patients with hip joint replacement could significantly relieve swelling and pain. It is helpful to improve the prognosis of patients and accelerate the rehabilitation process of patients. It is of great significance to the establishment of a good and harmonious doctor-patient relationship. It was helpful for the patients to recover the function of knee joint after operation and it was worthy of clinical application.

However, due to the limitation of our time and experience, the sample size collected is small, and there is no in-depth use of SAS scale to study the postoperative mood of patients, which is the shortcomings of this study. We expect that future scholars can combine SAS scale to obtain postoperative emotion related indicators of patients, so as to improve the level of nursing service.

## Figures and Tables

**Table 1:** General Information of Cases.

Groups	Cases	Average age	Body mass(kg)
Observation group	33 males	73.24 ± 3.32	62.21 ± 2.65
	29 females		
Control group	39 males	74.29 ± 3.35	62.25 ± 2.36
	23 females		

**Table 2:** Results of knee circumference diameter.

Groups	Cases	1d after operation	3d after operation	7d after operation
Observation group	62	29.71 ± 3.06	21.47 ± 2.29	14.26 ± 1.35
Control group	62	30.32 ± 3.34	25.34 ± 1.83	19.52 ± 1.91

**Table 3:** Results of knee pain.

Groups	Cases	1d after operation	3d after operation	7d after operation
Observation group	62	6.18 ± 1.33	3.32 ± 0.62	1.44 ± 0.36
Control group	62	6.14 ± 1.09	4.65 ± 0.85	2.69 ± 0.72

**Table 4:** Results of knee function.

Groups	Cases	1week after operation	1month after operation	3months after operation	6months after operation
Observation group	62	61.82 ± 3.52	71.26 ± 3.91	84.52 ± 4.21	93.70 ± 5.35
Control group	62	48.63 ± 3.06	62.13 ± 3.29	70.25 ± 3.66	81.64 ± 5.04

**Table 5:** Result of agitation situation.

Groups	Cases	Normal	Mild agitation	Moderate agitation	Severe agitation	Agitation rate
Observation group	62	60	1	1	0	3.23%
Control group	62	52	6	2	2	16.13%
*x^2^*	—	—	—	—	—	3.880
*P*	—	—	—	—	—	< 0.05

**Table 6:** Result of sleep time.

Groups	Cases	Pre-operation	Operation day	1d after operation
Observation group	62	4.23 ± 0.61	5.33 ± 0.62	6.01 ± 1.03
Control group	62	3.62 ± 0.75	3.97 ± 0.71	4.74 ± 0.91
*x^2^*	—	5.364	9.602	7.623
*P*	—	< 0.05	<0.05	< 0.05

## Data Availability

The datasets used during the present study are available from the corresponding author upon reasonable request.
